The article "Customer Experience towards the Product during a Coronavirus Outbreak" was retracted in 2023. Reasons: signs of a paper mill; suspected computer-generated content; unreliable results or conclusions; concerns about the data.

# Customer Experience towards the Product during a Coronavirus Outbreak

**DOI:** 10.1155/2022/4279346

**Published:** 2022-02-02

**Authors:** Sobia Wassan, Tian Shen, Chen Xi, Kamal Gulati, Danish Vasan, Beenish Suhail

**Affiliations:** ^1^Business School, Nanjing University, China; ^2^School of International Education, Nanjing University of CM, China; ^3^Amity University, Noida, Uttar Pradesh, India; ^4^Stratford University, Virginia, USA; ^5^School of Software, Tsinghua University Beijing, China; ^6^School of Economics, Shanghai University, China

## Abstract

Nowadays, sentimental analysis of consumers' review is becoming much crucial in the marketing world. It is not just giving ideas to the firms that how consumers like their product or service, but it would also help them make their service better. In this article, the statistical method identifies the relationship of many factors in consumer feedback. It introduces a deep-based learning method called DSC (deep sentiment classifier) to determine whether or not to recommend the reviewed product thoroughly. Our suggested method also investigates the effect sizes of the feedback, such as positives, negatives, and neutrals. We used the women's clothing review dataset containing 22,642 records after preprocessing of the results. Experimental studies show that the recommendations are an excellent positive sentiment indicator. In comparison, ratings become fuzzy performance metrics in product reviews. The 10-fold cross-validation analysis shows that the recommended form has the top F1 score (93.56%) in the sentimental classification on average and the recommended classification (88.32%) on average. A comparative description of other classifiers focused on machine learning, for example, KNN, random forest, logistic regression, decision tree, support vector machine multilayer perceptron, and naïve Bayes, also demonstrates that DSC gives the best possible result. We have tested DSC on the dataset IMDB (Internet Video Database), which includes the sentiment of the 50,000 movie reviews (25000 for training and 25000 for testing). In comparison to other baseline methods, DSC obtained an excellent classification score for this experiment.

## 1. Introduction

The study of emotions is a tactic of understanding the ideas, feelings, and expectations expressed in the text feature or the level of a sentence in a given text [1]. Today, enterprises use sites such as Twitter, forums, and blogs as reliable platforms to understand their consumers' expectations and improve their services. Sentiment analysis has become an attractive research field for collecting and assessing thoughts, feelings, and behaviours from sources of language, expression, and datasets that tally to how people respond to a given problem or event [2, 3]. Understanding consumer preferences based on the results of sentiment analysis will boost the industry world [4].

Nowadays, text mining is one of the most considered problems in the area defined above, a technique used to manually or automatically classify text. To address this gap, many studies have been investigated using sentiment analysis to interpret the comments found in chat forums, social media, and review pages [5–7]. Companies have frequently used the task described above to understand investors through their social media customer service teams.

In particular in e-commerce review analyses, there are three crucial approaches for assessing sentimental analysis:

- Lexical analysis
- Machine learning-based analysis
- Hybrid analysis

*Lexical analysis*: this method of categorizing the words of the response stream in their sections of expression and their reciprocal tagging, well known as POS tagging, is lexical analysis. It is a pretrained lexicon that is prepared for the method [8, 9].

*Machine learning-based analysis*: artificial intelligence is a subset of machine learning [10, 11] that is used for intelligent algorithms to train a correct classifier model. The research comprises preprocessing data, feature extraction, feature selection, testing, and labelling of the test dataset [12–14]. Deep learning methods are classified into three main classes: unsupervised learning, supervised learning, and semisupervised learning [1, 15, 16].

*Hybrid analysis*: hybrid methodology is a grouping of classification and regression problems. This methodology is more rapid and more precise than the other methods stated above.

In this article, on this dataset, we established a DSC for sentimental analysis and concentrated on the relationship of different factors in consumer reviews using statistical analysis, which included multivariate distributions, univariate distributions, multivariate analysis, and descriptive statistics [17]. During the first phase, we scrutinized the not-text feedback features (e.g., clothing, department name, ages, classes, and names) and the consumer references present in this dataset to analyze their relationship. We used a deep learning technique [18] to identify customer reviews' feelings about the products and assess whenever a positive review has been done for the purchased items. Generally, the main contributions of the present research work are as follows:

- Have a critical overview of similar studies on the study of sentimental analysis of consumer product review
- The way to examine the correlation between the different variables in the consumer product review depends on the four statistical research methods, containing multivariate distribution, univariate distribution, multivariate statistical analysis, and descriptive analysis
- Create a new deep learning algorithm called a deep sentiment classifier that accepts binary forms of text mining problems, such as a recommendation classification and a sentimental analysis on consumer review of purchased products
- Our method can automate the mining and selection of features. This methodology differentiates our contribution from that of [19–21] utilizing hand-crafted features
- Doing a comprehensive survey by performing several machine learning and conventional natural language and deep learning methods on these complex data to provide businesses with an understanding of how consumers like their goods and amenities

This paper is structured into sections: Section 2 presents the related work, Section 3 provides a list of the dataset used in this research, Section 4 set out realistic scientific work, Section 5 presents the conclusions as well as the discussions, and Section 6 concludes with several recommendations for future research.

## 2. Literature Work

Sentimental analysis is a type of data mining. We relied on predictive analysis and machine learning customer reviews of women's apparel e-commerce datasets. Some traditional methods focus on complex feature models or hand-crafted dictionary-based approaches for predictive analysis and sentiment analysis. In this article, we discussed the previous work on sentiment analysis. Authors [22] performed a hypothetical level of sentimental analysis. The researchers' focus is on three different lexicon techniques, supervised learning and unsupervised learning. At this time, we implemented supervised learning since we had access to supervised machine learning approaches and supervised data. That performed better than the unsupervised ones. Authors [23] addressed the tree-CRF approach to support binary and sparse function presentations. This methodology was a comprehensive and dynamic model of information.

In other words, [24] recommended a stacked denoising autoencoder technique that used a distributed feature to use such distributed word representations. That methodology outperformed tree-CRF as it could not provide a dynamic future structure and can be applied to many other domains. Tang et al.'s [25, 26] sentiment classification was implemented on microblog. Previously, authors used distributed word presentation as polarization, and scholars including [27] applied deep learning approaches. Their implementation was built using a single-layer CNN, while our method includes RNN and addresses two kinds of textual classification problems.

In some researchers [28, 29], a recursive autoencoder approach has been used to embed lexical information into deep learning. [8] proposed a Japanese emotion classification method that used a bidirectional long-term memory (LSTM) RNN network. After, it would be seen that integrating POS tag, word embedding, and Japanese polarization dictionary features strongly affected classification accuracy.

Authors [30] used the long-term memory system (LSTM) bidirectional recurrent neural network (RNN) to suggest and identify sentiments on datasets of e-commerce review. The results have shown that the recommendation is now a high positive sentiment metric. The bidirectional LSTM model mentioned above obtained an F1 score of 89% for the recommendation classified and 94% for the sentimental analysis. At the same time, our proposed model gained an F1 score of 89.32% for classifying recommendations and of 94.52% for classifying emotions.

Much like our proposed methods, Mousa and Schuller and Song et al. [31, 32] have built approaches using a bidirectional LSTM model to produce high-level information through expression and Asian consumer review datasets. In our study, we found actual consumer reviews on women's apparel for dataset analysis and used a deep learning method for sentimental analysis. This research applies natural language and machine learning methods to define large patterns in customer behaviour in text. In the data collection, the total number of unique words is 9811.

Our crucial objective existed to find out what consumers like and do not like about their purchasing. To accomplish this goal, we have performed observational analyses on this massive dataset. Firstly, we used to have to identify the features of the selected attributes and accelerate the difficulty of the analysis until a proper objective had been envisaged. And after that, through our research, we have shown that our statistical experiments are conducted using natural language methods. The results of sentiment analysis provided by state-of-the-art deep learning techniques have been considerable and helpful to e-commerce.

## 3. Material

- We used two distinct types of data sources in this analysis
- The sentiment of women's clothe e-commerce product review
- Movie review thought (IMBD) (Internet Movie Database)
- The sentiment of the women's clothe e-commerce product review dataset [17] is made by actual customers and is thus anonymized; i.e., brand names are replaced by suppliers and customer names are exempted. The data consisted of 22,641 user reviews with 9 supporting attributes, such as age, department, class name, and positive feedback count.  Table 1 describes the additional features with the titles, and Table 2 describes the frequency distribution and labelling of the features present in the dataset, such as age and recommendation ID

An analysis of IMDB's (50,000) movie reviews was performed using two positive features, text analysis, and sentiment analysis [5]. Compared to the previous benchmark functions, this framework gives considerably more information about quantitative emotion classification. The dataset includes a collection of 25,000 vastly polarized film reviews for preparation and 25,000 for analysis.

## 4. Technical Method

The computational method is distributed about three portions to evaluate the classification of sentiments: statistical analysis, deep learning, and machine learning analysis.

### 4.1. Statistical Analysis

The statistical analysis describes the computational relationship among variables using equations or models [33]. In this part, the dataset was analyzed using four statistical analysis methods, such as univariate distributions, multivariate analysis, multivariate distributions, and descriptive analysis. Drawing the plot was done using the author's text in [34].  Table 3 describes the statistical detailed info of the datasets.

#### 4.1.1. Analysis Univariate Distribution

*Age and positive feedback count distribution*: Figure 1 shows that most consumers aged 36-45 years had the most positive review of the products purchased. We also noticed two points from this analysis: (i) at the time of the analysis, e-commerce should include an emphasis on managing this section for the aged listed above, which remains with the utmost positive reviews, and (ii) electronic commerce will see that most of an age group remains quite pleased compared to more pleased age group of 36-45 years.

*Division name and department distribution*: Figure 2 indicates the frequency distributions of consumer ratings by division and department names.

*Distributions of division name*: the distribution of division names has three categories of standard, limited, and personal. This provided some perception into the size of the consumers' clothing sendoff comments.

*Distribution of department name*: this is important to remember that skirts and tops seem to be the most highly rated product. It will be fascinating to explore the motivation for leaving the analysis in the first place.

*Clothing ID distribution*: Figure 3 displays the top 60 IDs for clothes to identify the product's interest. Three dress IDs from 1079, 862, and 1095 have obtained considerably more ratings than others. As shown in Table 4, these products expected an average rating of 4/2 and an overall recommendation ratio of around 82%. They also observed that these products mainly were regular.

*(1) Distributions of Rating, Recommendation, and Label*. *Rating distribution*: the increasing number of ratings, with a score of five out of five, has been very positive. This proved that the department store was doing pretty well.

*Recommended IND distribution*: this factor represented the positivity of the rating distribution; however, as previously discussed, we assume that it produced the difference in positive thinking that had been societal rather than private.

*Label distribution*: we are surprised to find that the items were rated as three or better and recommended by the consumer. We predicted the relationship between rating and recommendation to be multivariate.

To figure out how customers express their hatred, we found these three variables especially promising. We based on the correlations between these variables in the multivariate section. The distribution of scores, recommendations, and labels is seen in Figure 5.

*Length of word*: Figure 6 indicates that the analysis's character and word counts are strongly correlated. They were equal in length, as seen in Table 5. The term and character count correlation coefficient are 0.99.

#### 4.1.2. Multivariate Distribution Analysis

*Division name by the department*: Figure 7 indicates that the general-sized top was the most dominant commodity. The dominance of general size within the department name was consistent across multiple categories, as seen in Figure 8. There had been a significant overall difference in the name of the general petite and the department.

*Name of class by department name*: Figure 9 provides a better look into the classification of multiple clothing types. As seen in Figure 10, the superiority of dress popularity was visible till now.

Figure 11 indicates that the most reviewed clothing styles were general-sized blouses, skirts, and knits, and Figure 12 indicates that most reviews have stayed popular for dresses with general petite sizes.

*Age as per positive feedback count*: Figure 13 indicates that age was marginally correlated with positive feedback counts. Focusing on the textual anatomy of incredibly positive reviews will be fascinating.

*Department and division naming recommendation*: the same observations are shown in Figure 14 as those found in Figure 7.

*Division and department rating names*: Figure 15 indicates that the division and department are compatible with the overall rating distribution.

The positive response count is under 40 through recommended IND and rating. This plot offers still more nuance only as a follow-up to a previous review of the dominant strongly positive reviews recommended by consumers. The first was a bump to the lower left: cutoff = true and recommended IND = 0.0. This strategy interacted unexpectedly with criticism of individual items; that is why the second bump (rate = 1) of the lighter blue dominated the positive feedback range of ~110. In the bottom-right plot, later performance was identified, while standard ratings were recommended. The vast range of yellow distributions with a ranking of 3 was interesting to see. Positive reviews of constructive criticism were the most highly rated. Also, see Figure 16 for more visualization.

*Rate by recommendation*: Figure 17 shows that five-star ratings are not preferred, but some cases recommend low-quality items. The recommended portion of the feedback for the more real instance of recommended and nonrecommended items with three scores is interesting to listen to, which could shed light on the utmost essential constraints on the store manager and the consumer's apparel behaviour.

#### 4.1.3. Descriptive Multivariate Analysis and Statistics

*Classification average by recommendation*: Figure 18 evaluates the rating recommendations. When recommended or reduced by the reviewer, the rating was below the maximum, so experimentation is not recommended. This process in the department and division has been persistent.

*Average ranking and recommended IND correlated by clothing ID*: Figure 19 shows the correlation between ratings and the dress ID recommended by IND. This heat map correlation indicates no relation between counts and average score, suggesting that the item's reputation did not contribute to special consideration once it came to average ratings. The age variables demonstrated similar behaviour.

However, there has been a high positive correlation of 80% between the recommended IND average and rating. A more quantitative view of the interest rate relationship is given in Figure 20 and focuses on the *p* value. The dots on the bottom left are the items that, in the expectation of maintaining the brand's reputation, definitely require attention from marketers.

*Class name average rating and recommended IND correlation*: in several class groups, Figure 21 shows significant relationships between average age and likelihood of recommendation.

### 4.2. Machine Learning Analysis

We use state-of-the-art machine learning classifiers for the role of emotion classification in this section, like naïve Bayes [35], KNN [12], support vector machine [36], random forest [37], logistic regression [38], decision tree [39], and multilayer perception [40]. We also considered both of these to be similar to the current DSC algorithm as simple classification methods.

The women's apparel dataset, which contains more than 23,000 user ratings with 9 attributes after preprocessing, was discussed during our first experiment (see Section 3). We reached an accuracy of 77.45% for KNN, 78.34% for RF, 73.34% for DTC (decision tree classifier) for this experiment, 77.25% for SVM (support vector machine), 82.80% for naïve Bayes, 82.75% for LR (logistic regression), and 82.80% for multilayer perceptron (MLP). The experimental findings show that the strongest classifiers for LR, naïve Baseline, and MLP remain with an accuracy of more than 80% across all these machine learning baseline classifiers.  Table 6 summarizes the complete results.

Our next experiment discussed the IMDB dataset, containing 50,000 sentiments for movie reviews (see Section 3). For this study, DSC remains outstanding with an F1 score of 88.64% among the simple classification methods, including linear regression, random forest, decision trees, naive Bayes, multilayer perceptron, SVM classifiers, and KNN (see Table 7).

### 4.3. Deep Learning Analysis

#### 4.3.1. Preprocessing

*Embedding and tokenizer*: for the analysis of documents, a fully convolutional neural network cannot be used directly; therefore, we must translate it somehow. There were two stages in the integration process. The first move was called a “tokenizer,” which translated text analysis from word to integer and was performed on the datasets before a neural network input [41]. The 2^nd^ phase had been an integral component of a neural network itself, called the “embedding” layer [42].

#### 4.3.2. Dropout

Dropout layers offer an optimal process to prevent overfitting, which can be accomplished by arbitrary dropout to ignore these neurons in the training point [43]. Because this helps to minimize codependent neuronal learning, we boost DSC dropouts with linear and exponential growth.

#### 4.3.3. Deep Sentiment Classifier

We introduced a deep sentiment classifier to extract a review text from the input series at numerous time phases. The recommended solution (DSC) is seen in Figure 22. The system was initially developed of the recurrent unit (RU) which has been internally set to 1 by TensorFlow each time a new series has begun. During the first phase, the word “this” is inserted into the RU that was used for its embedding layer (coded to zero) and also its gate to estimate a novel state. RU used another gate to measure the performance, but that was skipped since it simply included a description at the end of the series. In the 2^nd^ phase, the expression “is” was introduced into the RU that used the embedding layer that had been shifted by seeing all previous words “this.” There is no meaning in the term “this is” because by seeing these words, the RU probably did not save anything significant from its internal state.

Nevertheless, whenever the third word “not” was detected, RU discovered that the overall sentiment of input text could be valuable to calculate and therefore need to be recorded in the memory state of RU that can be used later once RU had seen the phrase “good” in step 6. Thirdly, RU generated a vector of values after the entire series was evaluated, summarizing what it should have found in the time stage. To obtain a goal node between 0.0 and 1.0, which has been understood either negatively (values near to 0.0) or positively, we have used a fully associated layer with activation of a sigmoid (values relative to 1.0). Two types of text classification problems were applied to the recommended classification model.

*Sentiment classification*: sentiment on consumer ratings of the product purchased is classified. In this dataset, the product analysis has negative, positive, and neutral feeling states. As a multinomial classification problem, we considered this type of problem.

*Classification by recommendation*: this identifies whether the product reviewed is recommended by the customers' reviews. Here, the product evaluation in the datasets contains two recommended and not recommended approval states. We found these types of issues to be binary classification problems.

## 5. Experimental Results and Discussion

### 5.1. Execution Environment

To evaluate our model in python3, we used TensorFlow [44], scikit-learn [45], and Keras [46]. Intel Core i5 2.67 GHz and 8 GB RAM are the computer systems used for this work. With the first learning rate of 0.0001, we used the Adam Optimizer.  Table 8 shows the setup of the parameter method proposed. During the training and testing of the proposed deep sentiment classification model, 10 k cross-validations were applied. For both recommendation and sentiment classifications, the average preparation, consistency testing, and loss by the deep sentiment classifier are discussed in Table 7.

### 5.2. Evaluation Metrics

We use the usual metrics to measure the efficiency of the classifiers [12, 47–49]: true negative (TN) is the correct negative review analysis, true positive (TP) is the correct analysis of a positive review, and fake positive (FP) means the positive test's false positive interpretation. The accuracy, precision, recall, and *F* measurement are determined using the gauges set out directly above. Accuracy is calculated as the proportion of all forecasts to the sum of the correct forecast results (see equation (1)). Precision indicates whether the model's positive predictions are accurate and are computed by dividing all positive predictions by the total number of true positives (shown in equation (2)). The recall is the positive described by the all feasible positive models and is accomplished by dividing the true positive by the actual positive total (shown in equation (3)). Its weighted average of recall and accuracy was F1-measurement. The controlled *F* score or *F* measure is now the precision and recall confusion matrix, as defined in equation (4).

(1) $$\begin{array}{c} \text{Accuracy}=\frac{\text{TP}+\text{TN}}{\text{TP}+\text{TN}+\text{FP}+\text{FN}}, \end{array}$$

(2) $$\begin{array}{c} \text{Precision}=\frac{\text{TP}}{\text{TP}+\text{FP}}, \end{array}$$

(3) $$\begin{array}{c} \text{Recall}=\frac{\text{TP}}{\text{TP}+\text{FP}}, \end{array}$$

(4) F1=2XPrcesion∗RecallPrcesion+Recall.

### 5.3. Experimental Setup

The efficiency of our proposed method (deep sentiment classifier) was compared in our experiment with 7 state-of-the-art machine learning methods:

- Trained classification algorithm with the training dataset and testing dataset
- Trained decision tree (DT) classification model with the training dataset and testing dataset
- Trained random forest (RF) classification model with the training dataset and testing dataset
- Trained SVM (support vector machine) machine learning algorithm with training data and analyzed by testing data
- Trained LR (logistic regression) classifier with the training dataset and testing dataset and trained computational modelling algorithm called multinomial (naïve Bayes) with training data and analyzed by the testing dataset
- A neural network model called MLP (multilayer perceptron) has been trained with training data and analyzed with test data

We compared the performance of our proposed method to many current methods of computational intelligence based on problems of sentiment classification (see Table 9).

### 5.4. Result and Discussion

Our proposed DSC method obtained an average accuracy of 93.55% for sentiment classification tasks under the experiment described above.  Table 10 shows the performance metrics of a new DSC methodology and other unique classifications based on the women's clothing databases for emotion detection tasks. It has been demonstrated that in terms of accuracy, precision, recall, and F1-measure, the method produced outperformed all other simple classifiers. In our DSC process, the F1 score is 25.53% more reliable than the KNN and RF baseline classifiers, 22.53% higher than the DTC baseline classifier, 14.53% higher than the LR baseline classifier, 13.53% higher than the Naïve Bayes baseline method, and 28.53 and 14.53% points higher than the SVM and MLP baseline classifiers, respectively.

With the other baseline IMDB dataset classifiers, Table 10 presents the experimental effects of the proposed DSC process. The experimental results show that DSC remained highly high among all baseline classification methods, with an F1 score of 88.01%.

Based on the sentiment classification analysis, Table 11 assesses the recommended method for existing techniques. It clearly shows that the approach proposed has remained extremely high compared to other approaches discussed.

It should, however, be stated that there was a variance in the distribution of frequencies between recommendation and sentiment groups. For example, more recommended reviews were done in the women's clothing database because there were more positive attitudes than potential and neutral ones. It can be a challenge for the model because it boosts the bias against a class of high-frequency propagation. Statistical analysis for the classification of recommendations is provided in Table 12. As shown in the table, comparatively, the deprecated class of the recommended classification problem gave worse predictions.

In addition, on the IMDB dataset, we tested DSC, which has a balanced sentiment for film reviews (25,000 for positive and 25,000 for negative). For the role of sentiment classification, which gained an average F1 score of 88.01% (see Table 13), our outcomes found that the deep sentimental classifier model was implemented well under the assumption that samples were spaced randomly and unevenly in the datasets.

Table 14 describes our proposed DSC success metrics and reflects our observations on the stigma against the imbalanced community (the class with the maximum frequency distribution). The predictive utility of the proposed technique was moderately low for neutral and negative emotions, as stated in the tables.

Despite imbalances in the dataset, our empirical analysis provided the facts with relatively high predictive performance to support the recommendation and sentiment classifications. Our findings showed that the bidirectional gated recurrent unit (GRU) was acceptable and highly predictive for analyzing customer reviews. We also advocate employing the unidirectional RNN-LSTM and CNN for a fair comparison in the future work on the same classification problem to further validate this conclusion.

## 6. Conclusion and Future Work

Online reviews are becoming a forum for trust building-consumer buying trends and affecting them. There is a need to manage such a massive number of comments with such dependency and provide reliable reviews before the user. This article analyzed two different types of datasets to classify sentiments: “women clothing review” datasets, consisting of 22641 records and IMDB sample size, containing 50,000 sentiments from the movie reviews. Our study is aimed at exploring the correlation between the different variables in the statistical analysis datasets of the review and at constructing a deep learning algorithm for DSC (deep sentiment classifier). Our proposed method addresses two types of text classification problems: (ii) classification of sentiments by recommendation, which investigates whether customer ratings recommend the product reviewed, and (ii) classification of sentiment by calculating consumer reviews' sentiment values toward the purchased product. In our proposed model, there is no feature selection technique used. DSC, however, performed well in the emotional classification, with an F1 score of 93.52% in the recommended classification of the women's clothing dataset.

In addition, on the IMDB datasets, we tested DSC, which has a balanced sentiment for film reviews (25,000 for positive and 25,000 for negative), which obtained an average F1 score of 88.01% for the task of data mining (see Table 12). Our results demonstrated which the model DSC worked well under the situation that samples in the dataset were spread uniformly and unevenly.

Furthermore, our analyses have shown that the recommendation is a reliable indicator for studying positive sentiment. Based on statistically analyses and state-of-the-art classifiers, our extensively investigated findings of this study will provide businesses with ideas on how to develop their services and satisfy consumer demands accordingly. On this model, many possible studies can still be performed. The tuning of hyperparameters for further development may be used in future works. The hyperparameters of the recommended method were restricted to one randomly selected parameter because of the computational cost limit.

## Figures and Tables

**Figure 1:** Customer age frequency distributions and positive feedback.

**Figure 2:** The frequency distribution per department and division of customer feedback.

**Figure 3:** Clothing IDs among the top 60 e-commerce apparel reviews.

**Figure 4:** The distribution of the frequency of the most tested classes of clothing.

**Figure 5:** The frequency distribution of rating, recommended IND, and label.

**Figure 6:** The distribution of count length and characters of the word.

**Figure 7:** The cross-tab demonstrates the superiority of the general-sized top.

**Figure 8:** Standardized cross-tabulation of clothing by department and division.

**Figure 9:** The domination of dress between clothe types.

**Figure 10:** Dress supremacy between types of clothing (class name by division name).

**Figure 11:** The types of clothing often reviewed, such as skirts, general-sized blouses, and knits.

**Figure 12:** The most reviewed clothing are from a standard petite size.

**Figure 13:** A slight relationship between ages and positive response cluster in a review.

**Figure 14:** Percentage of recommendation metrics per analysis by division and department.

**Figure 15:** The continuity in the distribution of rating shows.

**Figure 16:** The positive opinion obtained by more than 40 reviews and ratings.

**Figure 17:** A review rating expresses the recommendation status.

**Figure 18:** The improvement of recommendations and ratings.

**Figure 19:** The heat map showing the correlation between recommended IND by clothing ID and rating.

**Figure 20:** Rating and recommended mean by clothing ID.

**Figure 21:** Good correlations between both the average age and the probability of recommendation in different class groups.

**Figure 22:** Deep sentiment classifier model.

**Table 1:** Features available with description and data type in the women's clothing dataset.

Feature	Description	Type
Clothing's ID	Unique ID	int64
Ages	Reviewer ages	(int64)
Titles	Review titles	(Object)
Reviews	Reviews	(Object)
Rating	Reviewer rating on the product	(int64)
Recommended ID	Product is recommended or not	(int64)
Positive feedback count	Number of positive feedbacks	(int64)
Division name	Division name of the product	(Object)
Department name	Department name of the product	(Object)
Class name	Product type	(Object)

**Table 2:** Frequency distribution in women's apparel datasets of selected features.

Features	Unique counts
Clothing's ID	1173
Ages	78
Titles	13985
Text review	22622
Ratings	4
Recommended ID	3
Positive feedback counting	83
Division names	4
Department names	7
Class names	20

**Table 3:** Description of statistical analysis for women's data of clothes.

Feature	Mean	Std	Min	25%	50%	75%	Max
Clothing's ID	921.685909	203.683805	1.01	862.0	936.01	1078.0	1205.01
Ages	44.292881	13.328177	18.1	35.1	42.1	53.0	98.01
Ratings	42193093	1.125912	1.01	4.1	5.1	5.1	5.1
Recommended ID	0.828765	0.395223	0.01	1.1	1.1	1.0	1.01
Positive feedback count	2.641785	5.797521	0.01	0.1	1.1	3.0	123.01
Word counts	60.221951	28.543054	2.1	37.1	59.1	88.0	116.01
Character counts	308.771535	143.944127	9.1	187.1	302.1	459.0	509.01
Labels	0.885264	0.307223	0.1	1.0	1.0	1.0	1.0

**Table 4:** A clothing ID summary of statistical descriptions (1078, 1094, and 862).

Feature	Mean	Std	Min	25%	50%	75%	Max
Clothing's ID	1016.4849	104.396023	863.0	8623.0	1079.0	1095.0	1095.0
Ages	43.7249	13.150428	19.0	35.0	42.0	52.0	98.0
Ratings	04.1893	01.104307	01.0	04.0	05.0	6.0	6.0
Recommendation IND	00.8185	01.385593	0.0	2.0	01.0	01.0	1.00
Positive feedback counts	02.8625	06.773022	0.0	0.0	01.0	4.0	99.0
Word counts	060.5913	29.731487	2.00	37.0	61.0	88.0	116.0
Character counts	311.8605	145.836159	17.00	188.0	306.0	468.00	505.0
Labels	00.9025	01.296833	0.0	1.0	1.0	1.0	1.0

*Class name distribution*: as we can see in Figure 4, in the frequency of distributions, the top 3 clothing types (skirts, knits, and blouses) have been the most reported.

**Table 5:** Character count of review vs. word counts of the women's clothing dataset.

Review	Count	Mean	Std	Min	25%	50%	75%	Max
Word counts	22,629.00	61.22	29.54	3.00	37.00	58.0	89.00	116.00
Character counts	22,629.00	309.77	144.94	8.00	187.00	303.0	458.00	509.00

**Table 6:** A description of the success metrics compared to baseline classifiers using the women's clothing dataset for the proposed approach.

Method	Accuracy (%)	Precision (%)	Recall (%)	F1 score (%)
KNN	77.45	65	65	65
RF	78.34	80	80	80
DTC	73.34	73	73	73
LR	82.75	88	88	88
Naïve Bayes	82.80	81	80	80
SVM	77.25	75	75	75
MLP	82.80	87	87	87
DSC	80.01	80	80	80

**Table 7:** Deep sentiment classifier on average training and testing accuracy and loss.

Class	Train Acc (%)	Test Acc (%)	Train loss	Test loss
Recommended classification	97.48	89.33	0.03001	0.5068
Sentimental classification	99.99	94.56	0.0025	0.5326

**Table 8:** Hyperparameters for the deep sentiment classifier.

Hyperparameters	Values
Embedding size	8
Bidirectional gated recurrent unit	01
Batch size	64
Optimizer	Adam
Learning rate	0.0001
Epochs	50

**Table 9:** A description of the performance metrics similar to baseline IMDB dataset classifiers.

Method	Accuracy (%)	Precision (%)	Recall (%)	F1 score (%)
KNN	64.09	64	64	64
RF	79.61	80	80	80
DTC	72.79	73	73	73
LR	87.67	88	88	88
Naïve Bayes	83.37	83	82	82
SVM	75.58	75	75	75
MLP	83.37	87	87	87
DSC	88.01	88	88	88

**Table 10:** DSC method obtained an average accuracy.

Method	Accuracy (%)	Precision (%)	Recall (%)	F1 score (%)
KNN	25.53	40	40	40
RF	22.53	38	38	38
DTC	14.53	31	31	31
LR	13.53	29	29	29
Naïve Bayes	28.53	45	81	81
SVM	14.53	31	31	31
MLP	13.52	31	31	31
DSC	93.55	93	93	93

**Table 11:** Summary of key performance indicators compared to existing methods based on sentiment classification.

Methods	Accuracy (%)	Precision (%)	Recall (%)	F1 score (%)
Data on merchant ratings [24]	93.62	92.22	94.80	93.49
Reviews on Tsukuba corpus [24]	84.62	90.18	88.18	89.17
Analysis of customer product SVM [46]	81.75	—	—	—
Consumer product review by naïve Bayes [46]	68.57	—	—	—
Decision tree of consumer product ratings [46]	81.25	—	—	—
Reviews from Amazon on unlock smartphone [48]	97	—	—	—
Info on women's clothe reviews [30]	92.84	93	93	93
DSC (deep sentiment analysis)	93.55	93.68	93.52	93.52

**Table 12:** Recommended classification and result metric usage on women's apparel dataset (deep sentiment classifier).

Class	Precision (%)	Recall (%)	F1 score (%)
Recommended (1)	94.98	94.97	94.10
Not recommended (0)	71.83	68.91	70.41
Average/total	88	88	88

**Table 13:** Performance metrics using the IMDB dataset (DSC) on sentiment classification.

Class	Precision (%)	Recall (%)	F1 score (%)
Positively (1)	88	91	88
Negatively (0)	91	87	88
Average	88	88	88

**Table 14:** Metrics using DSC for sentiment classification results.

Class	Precision (%)	Recall (%)	F1 score (%)
Positive (0)	97.46	97.49	76.48
Negative (1)	49.41	51.16	50.39
Neutral (2)	33.47	21.95	26.04
Average/total	93	93	93

## Data Availability

The datasets we used in this study are publicly available at the following links: (1) https://www.kaggle.com/nicapotato/womens-ecommerce-clothing-reviews and (2) https://www.kaggle.com/lakshmi25npathi/imdb-dataset-of-50k-movie-reviews.
